# *In silico* Prediction of Deleterious Single Nucleotide Polymorphism in S100A4 Metastatic Gene: Potential Early Diagnostic Marker

**DOI:** 10.1155/2022/4202623

**Published:** 2022-07-31

**Authors:** Aisha Farhana, Sangeetha Kothandan, Abdullah Alsrhani, Pooi Ling Mok, Suresh Kumar Subbiah, Yusuf Saleem Khan

**Affiliations:** ^1^Department of Clinical Laboratory Sciences, College of Applied Medical Sciences, Jouf University, Sakaka, Al-Jouf 72388, Saudi Arabia; ^2^Department of Biotechnology, Saveetha School of Engineering, Saveetha Institute of Medical and Technical Sciences, Chennai, India; ^3^Department of Biomedical Science, Faculty of Medicine and Health Sciences, Universiti Putra Malaysia (UPM), Serdang 43400, Malaysia; ^4^Department of Medical Microbiology and Parasitology, Universiti Putra Malaysia (UPM), Serdang 43400, Selangor, Malaysia; ^5^Centre for Materials Engineering and Regenerative Medicine, Bharath Institute of Higher Education and Research, Bharath University, Selaiyur, Chennai 600073, Tamil Nadu, India; ^6^Institute of Bioscience, Universiti Putra Malaysia (UPM), Serdang 43400, Selangor, Malaysia; ^7^Department of Anatomy, College of Medicine, Jouf University, Sakaka, Al-Jouf 72388, Saudi Arabia

## Abstract

S100A4 protein overexpression has been reported in different types of cancer and plays a key role by interacting with the tumor suppressor protein Tp53. Single nucleotide polymorphisms (SNP) in S100A4 could directly influence the biomolecular interaction with the tumor suppressor protein Tp53 due to their aberrant conformations. Hence, the study was designed to predict the deleterious SNP and its effect on the S100A4 protein structure and function. Twenty-one SNP data sets were screened for nonsynonymous mutations and subsequently subjected to deleterious mutation prediction using different computational tools. The screened deleterious mutations were analyzed for their changes in functionality and their interaction with the tumor suppressor protein Tp53 by protein-protein docking analysis. The structural effects were studied using the 3DMissense mutation tool to estimate the solvation energy and torsion angle of the screened mutations on the predicted structures. In our study, 21 deleterious nonsynonymous mutations were screened, including F72V, E74G, L5P, D25E, N65S, A28V, A8D, S20L, L58P, and K26N were found to be remarkably conserved by exhibiting the interaction either with the EF-hand 1 or EF-hand 2 domain. The solvation and torsion values significantly deviated for the mutant-type structures with S20L, N65S, and F72L mutations and showed a marked reduction in their binding affinity with the Tp53 protein. Hence, these deleterious mutations might serve as prospective targets for diagnosing and developing personalized treatments for cancer and other related diseases.

## 1. Introduction

S100A4 is a calcium-binding protein belonging to the S100 family of proteins and contributes to the metastasis of different cancer. The increased expression of the S100A4 protein is associated with poor prognosis in patients with various cancer types and is a predictive marker for colorectal and breast cancer [1–6].

S100A4 exists in intracellular and extracellular forms and possesses no enzymatic activity. However, it has been shown to interact with numerous tumor-related proteins promoting tumor progression through an increase in motility, invasion, apoptosis inhibition, and cancer metastasis through the induction of prometastatic activities such as angiogenesis stimulation [7–9]. The stimulation of S100A4 attracts immune cells to the cancerous regions and promotes cytokine and growth factor secretion towards the tumor niche. T-lymphocytes are stimulated by chemotaxis by forming a complex with PGLYRP1, resulting in lymphocyte migration through the CCR5 and CXCR3 receptors.

The two EF-hand calcium-binding domains (helix-loop-helix motif) are parts of the S100 monomer protein, in which the N-terminal EF-hand comprises 14 amino acids. This part attaches the calcium through weak carbonyl oxygen atoms present in the backbone. At the same time, the C-terminal end is composed of 12 amino acids and binds calcium through the side-chain and carboxylates oxygen with higher affinity [10].

A striking conformational change occurs after calcium binding to the protein, resulting in the disclosure of a hydrophobic binding pocket in each monomer. The interaction of the calcium with the monomeric molecule paves the way for the binding of the other intracellular or extracellular proteins [11, 12]. Upon dimerization, p53 binds with S100A4 resulting in the degradation of p53. The proapoptotic function of Tp53 is also modulated by the binding of the C-terminal transactivation domain with S100A4, which leads to a reduction in the concentration of Tp53 protein levels [13].

S100A4 acts as a metastasin, playing a role in tumor progression by interacting with proteins that include p53 tumor suppressor proteins, annexin, nonmuscle myosin, and liprin *β*-1 [13–15]. The mutations which result in deleterious or neutral types may impact the protein structure or function and gene regulation and their downstream interactions with other proteins [16]. Deleterious mutations represent the harmful effect on the health of the organisms influenced by many genetic alterations, resulting in the cancer phenotype leading to driver alterations or also as simply drivers. This influences the cancer-related pathways, resulting in the occurrence of the same genes and loci in different patients, whereas the neutral mutations are believed to show nonsignificant phenotypic changes to neoplastic cells [17].

Among the SNPs, 50% of the mutations are consequences of nsSNPs and are reported in autoimmune, genetic, and inflammatory diseases. The changes in the amino acids due to SNPs could alter the protein structures as reflected by the changes in protein dynamics, geometry, charge, hydrophobicity, and finally, the interaction of the protein with other proteins or factors.

Hence, in the present study, the deleterious nonsynonymous SNPs of the S100A4 gene were identified, and their structural and functional effects were analyzed *in silico*. The detection of these deleterious SNPs could help propose the development of personalized treatments.

## 2. Materials and Methods

### 2.1. Retrieval of nsSNPs

The information on nsSNPs was retrieved from the National Center for Biotechnology Information (NCBI) (https://www.ncbi.nlm.nih.gov/snp/?term=S100A4), and their respective protein sequences were retrieved from Uniprot (Figure 1). The information on SNP ID, residue alteration, and location were accessed and subjected to subsequent studies.

### 2.2. Identification of Deleterious SNPs

The bioinformatics tools SIFT (https://sift.jcvi.org/www/SIFT_seq_submit2.html), PANTHER (Protein Analysis Through Evolutionary Relationship) (https://www.pantherdb.org/tools), PolyPhen-2 (Polymorphism Phenotyping v2) (https://genetics.bwh.harvard.edu/pph2/), PROVEAN (https://provean.jcvi.org/index.php), and Predict SNP (https://loschmidt.chemi.muni.cz/predictsnp) were used to predict the deleterious nsSNPs [18–21].

### 2.3. Identification of nsSNPs in the Domains of Protein S100A4

The software InterPro (https://www.ebi.ac.uk/interpro/) was used to identify nsSNPs locations on protein S100A4 conserved domains. The motif region, domain prediction, and functional characteristics of the proteins were identified by this tool [22].

### 2.4. Evaluating the Effect of the nsSNPs on Protein Stability

The impact of the mutations on the structure and stability of the protein was investigated by the I-Mutant 2-056 (https://folding.biofold.org/i-mutant/i-mutant2.0.html) tool, and the data of nsSNPs protein S100A4 was submitted in FASTA format [23].

### 2.5. Analyzing Protein Evolutionary Conservation

The ConSurf (https://consurf.tau.ac.il) tool was employed to identify the evolutionary conservation of amino acids. The analysis was based on the phylogenetic relationships between homologous sequences [24] (Figure 2). The nsSNPS that were found to be highly conserved were used, listed, and analyzed further.

### 2.6. Structural Effect Prediction on Human S100A4 Protein

HOPE61 (https://www3.cmbi.umcn.nl/hope/) was utilized to predict the SNP's effect on the protein structure. The S100A4 protein with the UniProt Acc IDQ8WWW0 and 24 individual nsSNPs were used as input [25, 26]. The Swiss-PDB viewer (https://spdbv.vital-it.ch/) was utilized for the mutated protein model generation with corresponding amino acid substitutions. The 3D Missense mutation tool was used to estimate the solvation energy and torsion angle of the mutations on the predicted structures. It was compared with the wild-type sequence for the deviations [27, 28]. TM-align was used for the comparison of the native and mutated protein structures.

### 2.7. Post-Translational Modification Sites Prediction

The different post-translational modifications of the proteins at amino acids such as serine, threonine, and tyrosine were predicted by the tool NetPhos 3.1. A score of greater than 0.5 was obtained through analysis by NetPhos 3.1 predicted amino acid phosphorylation. The sites of ubiquitylation and SUMOylation were also predicted.

### 2.8. Detection of SNPs in miRNA Target Sites

The miRNA seed and target site in UTR regions were detected using the Poly miRTS database web server, and the transcript NM_019554 was used as a query sequence (https://compbio.uthsc.edu/miRSNP/). The chromosome location chr1(-):153516094-153518282 and the SNP rs IDs were submitted to the analysis server.

### 2.9. Molecular Docking

The molecular interactions between the S100A4 protein of the selected deleterious mutations and the target protein Tp53 were studied using AutoDock Vina and ClusPro v2.0. The binding energy and the interactions of amino acid residues between the mutant models of S100A4 protein and Tp53 protein were analyzed.

### 2.10. Molecular Dynamics Simulation CABS-Flex 2.0

The CABS-flex 2.0 web server (http://biocomp.chem.uw.edu.pl/CABSflex2/) was used to study the dynamic simulation of the mutant proteins. The simulation was carried out with the default parameters of 50 cycles for 10 ns and a 1.0 fixed global weight for the modeled protein complexes.

### 2.11. Correlation of Identified SNPs in the COSMIC Database

The identified SNPs of the S100A4 gene were also verified in the COSMIC database to comprehend their effect on different malignancies. The COSMIC database provides comprehensive information on the somatic mutations of human cancer and their distribution (https://cancer.sanger.ac.uk/cosmic). The gene S100A4 was confirmed by searching for the missense mutation.

### 2.12. Protein-Protein Interaction (PPI) Networks and Functional Annotation

STRING v11 (http://www.string-db.org) was used to construct an interactome map of the S100A4 genes screened with the key genes involved in the EMT Pathways (TGF-*β*, Wnt, Notch, and Hedgehog signaling pathways). The PPI network was constructed with the key genes involved in this pathway, such as TGF-*β*, Smad 2, Smad-3, ZEB1, Foxc-2, TWIST, Snail, slug, E-Cadherin, N-Cadherin, *β*-Cadherin, PTEN, P13K, AKT2, GSK 3*β*, STAT-3, Cyclin D1, C-myc, Survin, MUC-1, PRR–X1, ZNF488, VGLL4, and Gli 1, were curated and subjected to the interaction analysis. Cytoscape (version 3.6.1) was used to visualize the PPI network, and the pivotal nodes were recognized based on the connectivity degrees.

## 3. Results

### 3.1. SNP Annotation

The NCBI dbSNP database for S100A4 had 1718 SNPs data in which 55 in-frame deletions, 57 initiator codon variants, 1232 intron, 54 noncoding transcript variants, and 137 SNPs were missense SNPs. Those 137 SNPs were subjected to further analysis.

### 3.2. Identification of Deleterious nsSNPs

Four different *in silico* nsSNP prediction tools predicted 24 SNPs of the protein S100A4 as deleterious and damaging (Table 1). The SIFT scores, PANTHER scores, and polyphen2 scores with the other neutral 55 neutral mutations that were screened were compared.

### 3.3. Identification of nsSNPs on the Domains of S100A4

InterPro predicted the two functional domains of the protein S100A4 as EF-Hand 1 and EF-Hand 2. The deleterious nsSNPs identified by different *in silico* nsSNP prediction tools were further subjected to identification of their location on the two domains, namely EF-hand 1 and EF-hand 2.

### 3.4. Determination of Protein Structural Stability

The RI (Reliability Index) and free energy change values (DDG-Delta Delta G) were predicted by the I-Mutant tool. This helped us to analyze the stability changes represented in Table 2.

### 3.5. Evolutionary Conservation Analysis

The ConSurf Analysis was carried out for 101 amino acid residues of S100A4 identified as SNPs. The highly conserved and exposed residues with the functional characteristics were identified as M1, E6, Y19, S20, G24, L29, E33, E41, E63, N65, D67, E74, N81, and K101. The residues L5, F16, L29, L62, and F72 were highly conserved structural residues buried within the protein structure.

### 3.6. Impact of nsSNPs on Human S100A4 Protein Structure

Among the mutations, F72V, E74G, L5P, D25E, N65S, A28V, A8D, S20L, L58P, and K26N were highly conserved and exhibited an interaction with the calcium-binding domain, EF-hand 1 or EF-hand 2 domains. The deleterious mutations F72V and E74G were located within the EF-hand 2 protein and were demonstrated to disrupt the calcium ion interaction. In the deleterious mutation, D25E, the amino acid residue of the wild type is smaller than the mutant residue. Distinctively, in the N65S deleterious mutation, the change in the amino acid to serine has made the occupied site significantly smaller and hydrophobic. This mutation highly affects the structure and causes destabilization as it is situated in EF-hand 2. Additionally, it also leads to the loss of the cysteine bond. The mutations K26N and S20L were analyzed as examples presented in Figure 3.

Similarly, the mutation in A28V causes disturbance in the core structure of the domain as the mutant residues are buried. In A8D, the mutant residues are bigger and neutral, disturbing the domain core structure and binding properties. The impact of the other deleterious mutations is presented in Table 3.

### 3.7. Structure Analysis of Mutant and Wild Models

3D models were predicted for the 24 deleterious nsSNPs and compared with the wild-type model, which showed the solvation energy of −0.42 and the torsion angle of −1.10. The mutation showed a higher deviation in both the solvation energy and the torsion from the wild type.

### 3.8. Post-Translational Modification Site Prediction

The phosphorylation sites were predicted at the regions of 15T, 50T, 20S, 60S, 64S, and 80S sites, and only the 60S highly deleterious nsSNP was found. The ubiquitylation sites were located at 100K and 101K predicted by UBpred. SUMOylation sites were not observed in any of the predicted highly deleterious nsSNPs.

### 3.9. Detection of SNPs in miRNA Target Sites

The PolymiRTS database detected four sites for miRNA binding due to 5 SNPs in the UTR region, and the sites were predicted to be abolished by these SNPs. The results are presented in Table 4.

### 3.10. Molecular Docking

All the mutant models of S100A4 interacted with a very low binding affinity with the Tp53 protein, as observed in Clus Pro, which ranged from −564.4 to 670. Also, the deviation in the hydrogen bond interaction with the target was observed. The energy minimization through the Swiss PDF viewer revealed a larger scale of variation for all the mutants, but in specific E88G, the wild-type showed −6525 kJ/mol and the mutant exhibited −7625.542 kJ/mol. Also the differences in the energy minimization was observed for the other mutants S20L (−6371.678 kJ/mol; A8D (−6392.843 kJ/mol); A8V (−6264.361 kJ/mol); D25E (−6578.558 kJ/mol); E74G (−6390.220 kJ/mol; F72V (−6420 kJ/mol); L5P (6319.368 kJ/mol).

### 3.11. Molecular Dynamics Simulations

Root mean square fluctuation (RMSF) was determined by molecular dynamic simulations to understand the atomic level deviation of the mutant proteins in physiological conditions. The RMSF values of the mutant models E88G and D25E were lower than the wild-type model. In the mutant model, E88G, a decrease in the RMSF value was observed (1.0650) compared to the wild-type (1.540). In the mutant model, D25E, the RMSF (3.5130) was very close to the mutant model with a RMSF value of 3.650. The alteration in the RMSF conferred a loss of versatility in the protein's mutant structure, leading to changes in the dynamic behavior. More flexibility was observed between the residues 30 and 70 which significantly affected the stability of the protein .

### 3.12. Correlation of Identified SNPs in the COSMIC Database

The search in the cosmic database resulted in the identification of 4 hits with the following Ensemble IdsS100A4_ENST00000368714; S100A4_ENST00000354332; S100A4,ENST00000368716.8; S100A4_ENST00000368715 and reported 388 mutations. Further analysis of the missense substitution of the Ensemble IdsS100A4_ENST00000368714 resulted in the report of E88K in the COSMIC database among the screened 21 nonsynonymous SNPs. This E88K mutation has been identified as a somatic mutation reported in large intestine carcinoma and adenocarcinoma. The tissue distribution of sample 1 has been reported for this mutation, with the FATHMM prediction score of 0.82 being pathogenic [13].

### 3.13. Protein-Protein Interaction (PPI) Networks and Functional Annotation

16 nodes and 65 edges in the PPI network had a local clustering coefficient of 0.734. An enrichment *p* value of less than <1.0*e* − 16 with an average node degree of 8.12 was detected. S100A4 gene interacted with the TWIST1, SNAI2, CDH2, CDH1, ZEB1, and SMAD2 directly and also with the other interactors such as PTEN, C-MYC, MUCI, CCND1, AKT2, and TGIF-2. Some PPI network connections with the S100A protein, signifying known and predicted genes are indicated in Figure 5.

## 4. Discussion

S100A4 interacts with the tumor suppressor protein Tp53 in the various cancer pathways and with other transcription factors involved in the EMT pathways. Thus, the mutations in S100A4 could influence the biomolecular interactions with their target proteins due to their aberrant conformations and possibly affect their downstream functions [29–31]. Therefore, identifying the deleterious nsSNPs in S100A4 could help determine their influence, detrimental effects, and progression mechanisms of various cancers [32].

Among the 77 nsSNPs of S100A4 found in the NCBI database, we screened 56 mutations showing neutral effects and 21 significantly deleterious nsSNPs using the PROVEAN *in silico* SNP prediction tool. However, among the twenty-one mutations, rs147390231 (T39I), rs199505533 (G92A), and rs368160023 (E88K) were observed to be tolerated in the SIFT algorithm. Polyphen and PANTHER identified 21 nsSNPs as damaging mutations and, hence, these were reconfirmed and analyzed by different tools (Figure 1). The deleterious mutations predicted thus far in our study were further studied through the InterPro tool to identify the location of the nsSNPs on various domains present in S100A4. The 21 mutations were located in the protein's EF-hand 1 and EF-hand 2 domains. Five nsSNPs were positioned in the EF-hand 1 domain and nine nsSNPs in the EF-hand 2 domain, disturbing the interactions and calcium-binding properties (Figure 2).

Among the highly scored deleterious mutations, F72V, E72G, L5P, D25E, N65S, ASV, ASD, S20L, L58P, F89I, and K26N were found to be largely conserved and affecting the functionality of the protein (Figure 3). The mutation F72V located in the domain of EF-hand 2, disturbs the interaction of the protein with the calcium ion. In E72G, the mutant residue is smaller, neutral, and hydrophobic than the wild-type residue and subsequently influences the interaction with the metal ion, calcium (Figure 4).

Similarly, in the L5P mutation, the size difference of the mutated amino acid influences its structural interaction. The amino acid residue phenylalanine at position 5 occupies a larger space in the wild-type protein. It forms a hydrogen bond with phenylalanine at position 27 and a salt bridge with lysine at position 28, which is disrupted in the mutated protein. In the D25E mutation, the mutant fails to form bonds at the respective position, affecting the stability (Figure 4). Furthermore, in N65S, the mutant residue is smaller than the wild-type residue. The lack of cysteine bridge formation affects the protein stability in the mutant type, causing the loss of interaction, which produces a severe effect on the 3D structure of the protein. In the A8V mutation, the mutant residue is bigger and buried in the core in contrast to the wild-type residue (Figure 4). This greatly influences the multimeric interactions of the protein. Additionally, the wild-type alanine is located in an alpha-helix, which is changed to an unfavorable valine residue in the mutant disturbing the core structure of this domain and affecting the binding properties of the protein.

For the A8D mutation, the mutant aspartic acid is negatively charged and less hydrophobic than wild-type alanine. Thus, the mutation has introduced a bigger and more charged residue, disturbing the multimeric interactions and protein folding properties. In S20L, the mutant residue is bigger than the wild-type residue. This mutation causes the loss of hydrogen bonds in the core, resulting in the disturbance of the correct folding, which subsequently influences the protein structure and function in the EF-hand 2 domain. Likewise, for the K26N mutation, the size differences of the amino acid disturb the interaction with the calcium ion, which leads to the destabilization of the domain (Figures 3 and 4).

The F89I mutation being both deleterious and highly conserved has the mutant residue, isoleucine located in a domain important for binding of other molecules. The mutation could influence the interaction between two domains and the possible loss of external interactions was predicted. The smaller size of the mutant residues is too small to make multimer contacts which could also affect the functionality of protein.

As predicted by the I-Mutant tool, the observed deleterious mutations in S100A4 showed a decrease in stability and significant changes in the RI and free energy change values (DDG).

Protein structural stability is important to maintain the native structure and function of the proteins. The structural and functional parameters were estimated in this study based on the ΔG value. The energy minimization through the Swiss PDF viewer revealed a larger scale of variation for all the mutants. Still, specifically for E88G, the wild-type showed −6525 kJ/mol and the mutant exhibited −7625.542 kJ/mol. Also the differences in the energy minimization was observed for the other mutants S20L (−6371.678 kJ/mol; A8D (−6392.843 kJ/mol); A8V (−6264.361 kJ/mol); D25E (−6578 .558 kJ/mol); E74G (−6390.220 kJ/mol; F72V (−6420 kJ/mol); L5P (6319.368 kJ/mol). All the predicted SNPs showed a negative value, indicating the decrease in the stability of the structure and hence its becoming unfavorable due to its unfolded/misfolded state (Figure 4 and Table 2).

Furthermore, the mutant structures were subjected to molecular simulations, and the RMSF was estimated to evaluate their flexibility under varying physiological conditions. Limited fluctuations and flexibility represent the stable structural state [33]. The RMSF of atomic residues of the mutant models was considerably different from the wild-type, which inferred the decrease in the thermodynamic stability of the mutant models. This further could impair the structural stability and the functions of the proteins. As S100A4 interacts directly with the tumor suppressor protein Tp53 and the other interactors of the EMT pathway in cancer, it may have a profound effect on tumor suppression.

About 14 different miRNAs were identified in this study that have altered SNPs. These miRNA were reported to be modulated in different cancers, namely, hsa-miR-505-5p (human cervical cancer), hsa-miR-1827; hsa-miR-650 (colorectal cancer), hsa-mir-3612; hsa-miR-940(cervical cancer), hsa–miR-4695-3p; hsa-miR-4763-3p; hsa-miR-3128 (ERBB2/Her2 gene) [34–40]. However, these alterations have been observed at different sites in regions other than the nsSNPs regions of the S100A4 gene (Table 4). It is noteworthy that these miRNAs can be explored further through proper clinical trials as potential treatment strategies.

The search for these deleterious nsSNPs identified that the E88K mutation was associated with the carcinoma of the large intestine and adenocarcinoma tissue samples. This signifies that studying these mutations in clinical samples and analyzing their possible effects on the interaction of S100A4 with the other proteins sought through *in vitro* and *in vivo* studies may lead to possible therapeutic interventions.

S100A4 has been demonstrated in the development of an aggressive metastatic phenotype progressing into cancer and metastasis. Also, the poor prognosis of cancer has been correlated with the upregulation of S100A4 in tumor cells, and its expression has been regulated by other factors like *β*-catenin, epidermal growth factor, tumor necrosis factor alpha (TNF-*α*), and methylation [41, 42]. In addition to its role in cancer metastasis, S100A4 is also reported in various pathophysiologies such as inflammation, fibrosis, angiogenesis, and neuroprotection [43–45]. Except for the E88K which is associated with colorectal carcinoma, the deleterious nonsynonymous SNPs identified in this study through the COSMIC database could be further explored in the tissue samples of various cancers and in different physiological conditions. Hence, further interaction studies could also help design and facilitate rational drug designing through miRNAs and personalized treatment in patients.

## 5. Conclusion

Comprehensive bioinformatics analyses for the identification of the deleterious nonsynonymous mutations were performed for the S100A4 gene, which are reported to play a significant role in cancer and other pathophysiological diseases. In this study, twenty-four deleterious mutations were identified by Provean, SIFT, Polyphen, and PANTHER. The SNPs E88G, S20L, A8D, A8V, D25E, E74G, F72V, and L5P were highly conserved and interacted with the EF-hand domain of the protein, showing significantly higher energy minimization and structural instability, ultimately affecting the functionality of the protein. The E88K mutation identified by our analysis has been reported in the COSMIC database. We conclude that the plethora of mutations identified in this study can be explored in tissue samples of the various cancer types and physiological conditions to facilitate rational drug designing through miRNAs for personalized cancer treatment.

## Figures and Tables

**Figure 1:** Pie chart indicating the SNP distribution in the S100A4 gene as retrieved from the dbSNP database.

**Figure 2:** Evolutionary conservation of S100A4 produced by ConSurf. The conservation scale variations of the different amino acids are given in which ‘e' represents an exposed residue; ‘b' represents a buried residue; ‘f' is a functional residue that is highly conserved and buried; ‘s' is a structural residue that is highly conserved and buried.

**Figure 3:** Structural analysis of the human S100A4 protein. Figures (a) and (b) represents the structural alteration due to the changes in the amino acid residue N26 and 20 L respectively as analyzed by Project HOPE. The green color represents the wild-type residue and the red color is shown by the mutant residue. (a) K26N. (b) S20L.

**Figure 4:** RMSF Plots of different mutants in comparison with the wild type of S100A4 Protein. (a) E88G. (b) D25E. (c) S20L. (d) F72V. (e) Wild type.

**Figure 5:** Protein-Protein interaction of the genes involved in different signaling pathways with S100A4 in String Database V 11.0. The colored nodes represent the first shell of interactors, and the green connecting lines represent the gene neighbourhood. The black lines between the genes represent gene coexpression.

**Table 1:** Identification of deleterious SNPs in S100A4.

SNP ID	SNPs	PROVEAN score	PROVEAN	SIFT	Polyphen2	PANTHER
rs116208483	L62V	−2.733	Deleterious	Deleterious	Damaging	Damaging
rs147390231	T39I	−2.735	Deleterious	Tolerated	Damaging	Damaging
rs148291612	F72V	−6.655	Deleterious	Deleterious	Damaging	Damaging
rs199505533	G92A	−2.645	Deleterious	Tolerated	Damaging	Damaging
rs200099267	E74G	−6.630	Deleterious	Deleterious	Damaging	Damaging
rs368160023	E88K	−2.842	Deleterious	Tolerated	Damaging	Damaging
rs373367471	L5P	−6.050	Deleterious	Deleterious	Damaging	Damaging
rs377093845	D25E	−3.493	Deleterious	Deleterious	Damaging	Damaging
rs536309763	N65S	−4.491	Deleterious	Deleterious	Damaging	Damaging
rs566299932	A8V	−3.698	Deleterious	Deleterious	Damaging	Damaging
rs566299932	A8D	−5.420	Deleterious	Deleterious	Damaging	Damaging
rs576307674	R40W	−4.053	Deleterious	Deleterious	Damaging	Damaging
rs747430747	S20L	−5.594	Deleterious	Deleterious	Damaging	Damaging
rs747868513	V70A	−3.450	Deleterious	Deleterious	Damaging	Damaging
rs751051544	E88G	−4.461	Deleterious	Deleterious	Damaging	Damaging
rs754093018	K57E	−2.525	Deleterious	Deleterious	Damaging	Damaging
rs759858655	L58P	−5.658	Deleterious	Deleterious	Damaging	Damaging
rs762009722	A8S	−2.619	Deleterious	Deleterious	Damaging	Damaging
rs762542639	L62P	−6.701	Deleterious	Deleterious	Damaging	Damaging
rs762597174	D92V	−4.467	Deleterious	Deleterious	Damaging	Damaging
rs766589410	F89I	−5.246	Deleterious	Deleterious	Damaging	Damaging
rs772235092	E69L	−6.263	Deleterious	Deleterious	Damaging	Damaging
rs868262406	K26N	−4.593	Deleterious	Deleterious	Damaging	Damaging
rs899447674	F72L	−5.865	Deleterious	Deleterious	Damaging	Damaging

**Table 2:** Prediction of the effect of nsSNPs on protein stability by I-MUTANT 2.0.

SNP ID	Amino acid substitution	I-mutant	DDG	RI
rs116208483	L62V	Decrease	1.75	8
rs147390231	T39I	Decrease	1.09	5
rs148291612	F72V	Decrease	−3.56	9
rs199505533	G92V	Decrease	−0.83	2
rs200099267	E74G	Decrease	−1.65	6
rs368160023	E88K	Decrease	−0.82	7
rs373367471	L5P	Decrease	−1.152	7
rs377093845	D25E	Decrease	0.05	1
rs536309763	N65S	Decrease	−0.88	8
rs566299932	A8V	Decrease	−0.07	2
rs566299932	A8D	Decrease	−1.12	4
rs576307674	R40W	Decrease	0.20	3
rs747430747	S20L	Decrease	−1.05	1
rs747868513	V70A	Decrease	−2.17	9
rs751051544	E88G	Decrease	−0.74	6
rs754093018	K57E	Decrease	−0.43	5
rs759858655	L58P	Decrease	−0.43	8
rs762009722	A8S	Decrease	−0.82	8
rs762542639	L62P	Decrease	−2.32	7
rs762597174	D92V	Decrease	0.76	2
rs766589410	F89I	Decrease	−1.04	8
rs772235092	E69L	Decrease	0.08	4
rs868262406	K26N	Decrease	0.16	1
rs899447674	F72L	Decrease	−2.52	8

**Table 3:** Mutational effects on the structure and conservation of the S100A4 protein.

S.No	Mutation	Structure	Conservation
rs116208483	L62V	EF-hand -2	Not conserved
rs147390231	T39I	EF-hand 1	Not conserved
rs148291612	F72V	EF-hand domain	Located near a highly conserved protein
rs199505533	G92V	Surface of the domain	Not conserved
rs200099267	E74G	Surface of the domain	Conserved
rs368160023	E88K	Surface of the domain	Not conserved
rs373367471	L5P	Surface of the domain	Conserved
rs377093845	D25E	EF-hand 1	Very conserved
rs566299932	A8V	EF-hand domain	Very conserved
rs566299932	A8D	Surface of the domain	Very conserved
rs576307674	R40W	EF-hand 1	Not conserved
rs747430747	S20L	EF-hand 1	Very conserved
rs747868513	V70A	EF-hand 2	Very conserved
rs754093018	K57E	EF-hand 2	Conserved
rs759858655	L58P	EF-hand 2	Not conserved
rs766589410	F89I	EF domain hand pair	Very conserved
rs868262406	K26N	EF-hand 1	Very conserved
rs762542639	L62P	EF-hand 2	Very conserved
rs536309763	N65S	EF-hand 2	Very conserved
rs751051544	E88G	EF-hand 2	Not conserved
rs762542639	L62P	EF-hand 2	Very conserved
rs762597174	D92V	Present in turn	Not conserved
rs772235092	E69L	EF-hand 2	Very conserved
rs899447674	F72L	EF-hand 2	Not conserved
rs147390231	T39I	EF-hand 1	Not conserved

**Table 4:** Detection of SNPs effect in the S100A4 regulatory region by PolymiRTS database.

Location	dbSNP ID	Variant type	Wobble base pair	Ancestral	Allele	miR ID	Conservation	miRSite	Function	Experimental	Context + score change
				Allele					Class	Support	
153516154	rs113443697	**SNP**	**N**	**G**	G	hsa-miR-505-5p	7	acccTGGCTCCtt	D	N	−0.217
					C	hsa-miR-1207-5p	5	aCCCTGCCtcctt	C	N	−0.255
						hsa-miR-1827	5	accCTGCCTCctt	C	N	−0.169
						hsa-miR-3612	7	acccTGCCTCCtt	C	N	−0.216
						hsa-miR-4695-5p	5	accctGCCTCCTt	C	N	−0.238
						hsa-miR-4763-3p	5	aCCCTGCCtcctt	C	N	−0.255
						hsa-miR-650	7	acccTGCCTCCtt	C	N	−0.16
						hsa-miR-6808-5p	5	acCCTGCCTcctt	C	N	−0.189
						hsa-miR-6893-5p	5	acCCTGCCTcctt	C	N	−0.17
						hsa-miR-940	5	acCCTGCCTcctt	C	N	−0.133
153516160	rs1051044	**SNP**	**N**	**A**	**C**	hsa-miR-6798-5p	**6**	TtttcCCCCCTGg	**C**	**N**	−**0.226**
153516185	rs143742855	**SNP**	**N**	**C**	**C**	hsa-miR-1273a	**2**	cccTGTCGCCAgt	**D**	**N**	−**0.437**
					**T**	hsa-miR-196a-3p	**2**	cccTGTTGCCAgt	**C**	**N**	−**0.264**
					**T**	hsa-miR-3128	**2**	ccctgTTGCCAGt	**C**	**N**	−**0.093**

N in wobble pair column represents ‘No.' This indicates that the particular SNP cannot form a G:U wobble base pair with miRNA. N in the experimental support column also represents ‘No' It indicates that so far no experimental data have been reported for the predicted target site. In the functional class column, D represents that a derived allele disrupts a conserved miRNA site (ancestral allele with support ≥2), and N represents that the derived allele disrupts a nonconserved miRNA site (ancestral allele with support ≥2).

## Data Availability

Data used in this study are available as hyperlinks in this paper.
